# Pattern Recognition of Holographic Image Library Based on Deep Learning

**DOI:** 10.1155/2022/2129168

**Published:** 2022-02-18

**Authors:** Bo Wu, Changlong Zheng

**Affiliations:** ^1^Faculty of Education, Northeast Normal University, Changchun 130021, China; ^2^High School Attached to Northeast Normal University, Changchun 130021, China

## Abstract

The final loss function in the deep learning neural network is composed of other functions in the network. Due to the existence of a large number of non-linear functions such as activation functions in the network, the entire deep learning model presents the nature of a nonconvex function. As optimizing the nonconvex model is more difficult, the solution of the nonconvex function can only represent the local but not the global. The BP algorithm is an algorithm for updating parameters and is mainly applied to deep neural networks. In this article, we will study the volume holographic image library technology, design the basic optical storage path, realize single-point multistorage in the medium, and multiplex technology with simple structure to increase the information storage capacity of volume holography. We have studied a method to read out the holographic image library with the same diffraction efficiency. The test part of the system is to test the entire facial image pattern recognition system. The reliability and stability of the system have been tested for performance and function. Successful testing is the key to the quality and availability of the system. Therefore, this article first analyzes the rules of deep learning, combines the characteristics of image segmentation algorithms and pattern recognition models, designs the overall flow chart of the pattern recognition system, and then conducts a comprehensive inspection of the test mode to ensure that all important connections in the system pass through high-quality testing is guaranteed. Then in the systematic research of this paper, based on the composite threshold segmentation method of histogram polynomial fitting and the deep learning method of the U-NET model, the actual terahertz image is cut, and the two methods are organically combined to form terahertz. The coaxial hologram reconstructs the image for segmentation and finally completes the test of the system. After evaluation, the performance of the system can meet the needs of practical applications.

## 1. Introduction

Image denoising is to reduce the noise in the image, and the low-resolution image is transformed to form a high-resolution image organically is the image superresolution technology [1]. Both can effectively improve image quality without changing the existing hardware equipment and imaging process [2]. In recent years, deep learning technology has achieved substantial breakthroughs and developments, bringing about tremendous changes in many fields [3]. Deep learning technology is derived from the second generation of neural network technology, which deepens the ability to process data through a deep network structure [4]. In the image field such as image noise and image superresolution, deep learning technology is developing rapidly and has achieved processing effects far exceeding traditional image processing technology. Add the existing deep learning segmentation algorithm to the 2.52 THz coaxial holographic image library for simultaneous processing [5]. Although the number of training samples is insufficient, U-NET can still accurately segment the electron microscope neuron image. According to the experiment in this article, for the real terahertz coaxial digital holographic image library, reconstruct the insufficient number of samples and analyze the U-NET segmentation results of the training set, loss function, and learning rate that affect the real terahertz image, so that it gets the best model. The experimental results show that the optimized U-NET model has the specific ability to distinguish between the image target and the background and at the same time has a specific noise reduction function, which can eliminate the more serious noise in the image [6]. It is proved that in the experiment, the noise in the gear image is basically eliminated, and the target is better retained. The segmentation result is better than the combined threshold segmentation method, but the seal image must be segmented by other algorithms [7]. The powerful Visual Studio development tool completes the development of the facial image pattern recognition system, with a high-quality interface and excellent friendliness. In the process of designing the system software, the confidentiality and special functions of police cases are integrated [8]. The customer adopts modular thinking in the design process to more easily identify the identity of others. It is composed of several important modules and is a kind of user-friendly approach. The database is mainly used to provide the client with interface configuration information, user credentials, and standard facial images. The database deployment in the system research is mainly used to save user credentials and login time and to compare with the recognized images. The design process of this article selects the SQL2008 database based on the skill level of the security assessment and the system survey.

## 2. Related Work

### 2.1. DnCNN Network

The literature introduces the application of deep convolutional neural network of DnCNN model to image denoising in terahertz image. First, the principle of noise suppression related to the network structure of the DnCNN network is studied [9]. Then optimize the network model from the relevant parameters of the neural network to obtain the most suitable denoising network for terahertz images [10]. Then the traditional denoising algorithms of NLM and BM3D are introduced, and their related parameters are optimized. Finally, the denoising effect of the DnCNN network is compared with the traditional denoising algorithm, and the denoising effect of the deep neural network model in this chapter is analyzed and compared [11]. The literature introduces the application of densely connected networks in the image superresolution of terahertz images [12]. First, we will introduce the network structure based on tightly connected networks and the principles of high-resolution networks. Then optimize the network model from the relevant parameters of the neural network to obtain the most suitable superresolution network for terahertz images [13]. Then introduced the traditional superresolution algorithm based on sparse representation and anchored neighborhood regression and optimized its related parameters. Finally, the denoising effect of the superresolution network of the dense residual network is compared with the traditional superresolution algorithm. The literature introduces the traditional terahertz image segmentation method and its improved algorithm. The composite threshold segmentation technique is used to characterize the actual holographic reconstructed terahertz image [14]. This means that when trimming and mirroring, the surrounding background will be removed first, and then filtering and denoising will be performed [15]. After the image is improved by grayscale stretching, a polynomial fitting histogram will be performed for threshold segmentation, and the two threshold methods and the Otsu method will be compared step by step [16].

### 2.2. U-NET Segmentation

The literature introduces the compound U-NET segmentation algorithm. Based on the research of segmentation of the holographic reconstructed terahertz image based on the combined threshold segmentation method and U-NET segmentation algorithm, the trimming and mirroring expansion steps, the NLM filter processing the terahertz image, and then the U-NET segmentation, repeat the experiment to the segmentation result is enlarged, the influence of the existing random features is reduced and the target is better maintained. The literature introduces the U-NET segmentation algorithm as a deep learning algorithm for segmentation of holographic reconstructed terahertz images [17, 18]. The deep learning segmentation algorithm learns and understands data by simulating the learning method of the human brain and can understand the training data before processing any other data. It has been partially applied [19]. U-NET relies on data expansion in order to use training images more effectively and accurately segment electron microscope neuron images from very few training images. This will reduce the sample size of the actual coaxial digital holographic terahertz reconstruction in this experiment [20]. In the experiment, we optimize by comparing and analyzing the results to obtain a model of the actual terahertz image that is particularly suitable for the experiment [21].

After reading the above literature, it can be determined that the main work of this paper includes Figure 1nodes.

## 3. Deep Learning and Pattern Recognition Technology of Holographic Image Library

### 3.1. Principles of Deep Learning

Artificial neural network originated from the mathematical bionic modeling of human nerves. Modern artificial neural network models are an important part of machine learning and an important foundation of deep learning.

The output of a single neuron can be expressed as (1)

(1) $$\begin{array}{c} y=f\left(\sum_{i}^{n}w_{i}x_{i}+b\right). \end{array}$$

Artificial neural network fits the model through training, so as to achieve the purpose of learning. The training process of a single neuron can be expressed by (2). The network is trained by updating the weights each time the error between the network's predicted value and the true value. Among them, *k* represents the *k* training, *i* represents the *i*th data category, and *λ* represents the learning rate.

(2) $$\begin{array}{c} w^{\left(k+1\right)}=w^{\left(k\right)}+\lambda \left(y_{i}-{\hat{y}}_{i}^{\left(k\right)}\right)x_{i}, \end{array}$$

∂*C*/∂*w*_*i*_ and ∂*C*/∂*b*_*i*_ are obtained by the chain derivation rule.

(3) $$\begin{array}{c} w_{i}^{+}=w_{i}+\Delta w_{i}=w_{i}-\lambda \frac{\partial C}{\partial w_{i}},\\ b_{i}^{+}=b_{i}+\Delta b_{i}=b_{i}-\lambda \frac{\partial C}{\partial b_{i}}. \end{array}$$

The loss of the network is propagated backward step by step through the chain derivation process, and the value of the parameters of each layer of the network from the back to the front is changed, so that the network can be trained.

(4) $$\begin{array}{c} \frac{\partial C}{\partial w_{5}}=\frac{\partial C}{\partial {\text{Out}}_{o1}}\frac{\partial \text{ Out}{\;}_{o1}}{\partial {\text{Net}}_{o1}}\frac{\partial {\text{Net}}_{o1}}{\partial w_{5}}. \end{array}$$

The formula of mean square error (MSE) corresponds to (4). The characteristic of using squaring to calculate the error is that when the difference between yi and (xi) is greater than 1, the squaring calculation will increase the error, giving it greater punishment, and speeding up the training. And when the difference between yi and (xi) is less than 1, the square calculation will reduce its error, thereby giving it a smaller punishment, and making the training more accurate. But at the same time, MSE will also give higher weight to abnormal points, which will reduce the overall performance of the model and lead to phenomena such as overfitting.

(5) $$\begin{array}{c} \text{MSE}=\frac{1}{n}\overset{n}{\underset{i=1}{\sum }}{\left(y_{i}-f\left(x_{i}\right)\right)}^{2}. \end{array}$$

Mean absolute error (MAE), its mathematical expression is as (5), minimizes the absolute value of the error to train the model. Unlike MSE, the gradient of MAE is equal everywhere, which also means that MAE will still give the same punishment to small losses as large losses, which is not conducive to the efficient convergence and learning of the model. But at the same time, because MAE gives all errors the same weight, it is not as sensitive to outliers as MSE. Using MAE to calculate loss is more conducive to learning from data with fewer outliers.

(6) $$\begin{array}{c} \text{MAE}=\frac{1}{n}\overset{n}{\underset{i=1}{\sum }}\left|y_{i}-f\left(x_{i}\right)\right|. \end{array}$$

L0optimizer was proposed by Louizos C et al. in 2017. Its mathematical expression is as in (7), where the term *δ* is a constant term of a hyperparameter, and *δ* is taken as 10^−8^ in the algorithm of this paper.

(7) $$\begin{array}{c} L0\text{Loss}=\frac{1}{n}\overset{n}{\underset{i=1}{\sum }}{\left(\left|y_{i}-f\left(x_{i}\right)\right|+\delta \right)}^{2},\\ L0\text{Loss}=\frac{1}{n}\overset{n}{\underset{i=1}{\sum }}{\left({\left(y_{i}-f\left(x_{i}\right)\right)}^{2}+\delta \left|y_{i}-f\left(x_{i}\right)\right|+\delta^{2}\right)}^{2}, \end{array}$$

tanh is a hyperbolic tangent function, proposed by Malfliet et al. in 2005, and its function expression is as (7)

(8) $$\begin{array}{c} f\left(x\right)=\frac{e^{x}-e^{-x}}{e^{x}+e^{-x}}. \end{array}$$

But at the same time, the zeroing mechanism of the ReLU function also brings its shortcomings. If the back propagation process of the network (including the ReLU function) has large gradient fluctuations, the ReLU input distribution is concentrated in the almost negative area, then such A large number of negative inputs will cause a large number of outputs of the ReLU function to be 0. A large number of neurons are permanently closed because the gradient cannot be updated. This phenomenon is called Dead Relu. At the same time, unsuitable network parameter initialization methods, such as a large number of weights being initialized to 0, will also cause Dead Relu problems. Dead Relu can cause training problems such as vanishing gradients.

(9) $$\begin{array}{c} f\left(x\right)=\left\{\begin{array}{cc} x, & \text{if}x>0,\\ 0, & \text{if}x\leq 0. \end{array}\right) \end{array}$$

The ELU function was proposed by Clevert et al. in 2015. Its function expression is shown in (8)

(10) $$\begin{array}{c} f\left(x\right)=\left\{\begin{array}{cc} x, & \text{if}x\geq 0,\\ \alpha \left(e^{x}-1\right), & \text{if}x<0. \end{array}\right) \end{array}$$

PReLU was proposed by He K et al. in 2015. It is a variant function of the ReLU function. Its principle is the same as that of the Leaky ReLU function, which is to prevent the Dead ReLU problem in the ReLU function by giving a small slope to the negative input. But unlike the slope parameter in Leaky ReLU, which needs to be manually specified, the parameters in PReLU can be optimized through learning. Its function expression is as (9), where *λ* is a learnable parameter vector with the same shape as *x*.

(11) $$\begin{array}{c} f\left(x\right)=\left\{\begin{array}{cc} x, & \text{if}x>0,\\ \lambda x, & \text{if}x\leq 0. \end{array}\right) \end{array}$$

For a network that has not undergone batch normalization, take the sigmoid activation function as an example. If the data falls in the area with a small gradient, then the network may cause slow training due to the small gradient, or even cause the gradient to disappear. Training has stalled.

Use the mean and variance of each data batch to batch standardize the data to promote normal data distribution. The processed data are concentrated in the area with a large gradient at the center of the function.

However, the obtained normal distribution data may not achieve the best results. The gradient between the red dotted lines of the sigmoid function does not change much, so the effect of the non-linear transformation of the non-linear function cannot be reflected. Therefore, in the fourth step, the scale factor *γ* and the translation factor ß are introduced for batch standardization, which can be adjusted through training so that the network obtains the best distributed data. While preventing the gradient from disappearing, the non-linear function of the activation function is better utilized, which is more conducive to training.

### 3.2. Image Desiccation Algorithm

The DnCNN network is a deep convolutional neural network. It is based on the residual strategy used to remove noise from the image. It better solves the problem of neural network degradation caused by the gradient instability of the deep network and can be achieved at a deeper network depth—a stable convergence of the network under. It has achieved far more effects than traditional image denoising methods in image denoising [22].

The idea of the residual strategy mainly comes from the ResNet network. The ResNet network forms a residual block by adding a fast connection between every two convolutional layers to stabilize the gradient in the network. In the DnCNN network, the residual block design is not used, that is, the output of the network in the output layer is the noise part of the image [23]. And because the image and noise are additive, so to get the denoised picture, you only need to subtract the original picture from the noise picture output by the network. In the residual learning of ResNet, it can be proved that when the residual is very small, the layer-to-layer is close to the identity mapping, and the network at this time is very well trained. Therefore, in the DnCNN network, when the noise level is low, the error between the noise picture and the pure picture is also small, the network residual is also small, and the network training is simpler [24].

The simplified network structure of DnCNN is shown in Figure 2. In the DnCNN network, the main body of the network is the superposition of several identical convolutional layers. No pooling layer is added to the entire network. Each convolutional layer uses the “same” pattern to fill the edge of the feature map and ensures that the step size of each convolution kernel is 1 so that the size of the feature map is in the entire network keep constant. Except for the first and last convolutional layers, BN layers and activation function layers are added after each convolutional layer [25]. The number of convolution kernels in the termination stage of the convolutional layer is 1, and the purpose is to make the dimension of the final output tensor same dimension as the input image [26]. The final output of the network is the difference between the input image and the residual tensor of the last layer of convolution.

Using MSE as the loss function training network, its denoising result index is shown in Table 1.

The network trained with MAE as the loss function, the index of the denoising result is shown in Table 2.

Using Looptimizer as the loss function training network, the index of the denoising result is shown in Table 3.

### 3.3. Pattern Recognition Model of Holographic Image Library

Feasibility study is the first task at the beginning of software development. If the problem cannot be solved, time, resources, and human resources are all wasted on software development. Nowadays, the optical image document recognition industry model has formed a certain theoretical tone through the development of recognition theory and image processing technology. Optical character recognition (OCR) continues to develop based on optical image processing and has taken a place in various fields of social life. Optical character recognition has the advantages of high speed, high efficiency, low error, and low cost of text input. As a new technology, various fields of social life are inseparable from document recognition based on optical character recognition. The characters on the ID card are unique documents, and the development of ID card recognition technology based on optical images has matured [27]. Therefore, the ID card information recognition system based on optical images is technically feasible. Currently, most ID card information is obtained by identifying high-frequency information embedded in the ID card or manually inputting it. The manual input method is inefficient and error-prone, so it will not be possible to obtain photo information [28]. On the other hand, the radio frequency identification method requires the increase of radio frequency chips for system identification and related application development, which promotes the increase of equipment costs. The effective use of computer technology in today's society, comprehensive, effective, fast and cheap access to personal data, verification, and management has become an urgent problem in the current population information flow management [29]. This theme is a very large application value theme and has high requirements in the fields of public safety, transportation, and services. By designing and implementing an ID card recognition system based on image processing and pattern recognition technology, we can provide the responsible department with an effective, fast, and cheap method of inputting personal ID card information. This method can facilitate the inquiry and verification of identity information and further promote the network and computerization of government agencies. Improving the cost and labor efficiency of services and government departments has important practical significance [30].

Table 4 shows the histograms of the R, G, and B channels. The histogram divides the illumination of the image into four areas. The first range is 0–25. This area mainly contains the black background and the text information on the ID card, which is the area with low gray value. The second area has a range of 25 to 50 and includes ID-specific information such as “name,” “gender,” and “ethnicity.” The three channels in the third zone are slightly different, the blue channel is 50–120, and the red and green channels are about 50–150. The fourth is the remaining area with few pixels, which is the highlight area caused by uneven light in the image.

The image characteristic comparison table of the standard area and the highlight area is shown in Table 4. Comparing Table 4, it can be seen that in terms of gray mean, standard deviation, and average volatility, the standard area and the highlighted area are relatively close, but there is a big change in the average deviation. Therefore, by changing the average displacement rate, the highlight area of the ID card image can be corrected.

Define the average gray level of each channel as

(12) $$\begin{array}{c} \bar{I_{x}}=\frac{\sum_{x}N_{x}}{,}x=R,G,B. \end{array}$$

Define the gray volatility rate of each channel:

(13) $$\begin{array}{c} K_{x}=\frac{l_{x}}{I_{x}},x=R,G,B. \end{array}$$

Define the color shift rate of each channel:

(14) $$\begin{array}{c} {\text{Rate}}_{x}=\frac{I_{x}^{s}}{l_{x}^{d}},x=R,G,B. \end{array}$$

Use the highlight area shift rate to correct the highlight area. First, classify the light according to the intensity of the highlight area, calculate the average deviation rate of each layer, and correct the pixels with high gray values as follows:

(15) $$\begin{array}{c} I_{\text{xnew}}^{s}=\frac{l_{x}^{s}}{{\bar{\text{Rate}}}_{x}},x=R,G,B. \end{array}$$

The global threshold method uses a variety of algorithms to determine a threshold *T* that is independent of pixel position. Methods for determining the value of *T* include Otsu's method and iterative algorithm. The Ostu method is also called the maximum difference between classes. It provides automatic selection of *T* by counting the histogram attributes of the entire image. If the threshold between the two categories is *t*, then the two categories are C_0_ and C_1_:

(16) $$\begin{array}{c} C_{0}=\left\{0,1,\ldots t\right\},C_{1}=\left\{t+1,t+2,\ldots ,255\right\}. \end{array}$$

Then the Ostu method finds the maximum value of the following formula:

(17) $$\begin{array}{c} \eta =\frac{\sigma_{B}^{2}}{\sigma_{T}^{2}}. \end{array}$$

The Bresen algorithm mainly uses the median between the maximum and minimum values of each pixel area as the segmentation threshold.

(18) $$\begin{array}{c} C\left(x,y\right)=G_{\max}-G_{\min}<l. \end{array}$$

The new judgment criteria are as follows:

(19) $$\begin{array}{c} g\left(x,y\right)=\left\{\begin{array}{cc} 0 & f\left(x,y\right)<\left(1-\beta \right)T,\text{ or },\left(f\left(x,y\right)<T_{\text{Bn}}\left(x,y\right),\text{ and },\left(1-\beta \right)T\leq f\left(x,y\right)\leq \left(1+\beta \right)T\right),\\ 1 & f\left(x,y\right)>\left(1+\beta \right)T,\text{ or },\left(f\left(x,y\right)\geq T_{\text{Bn}}\left(x,y\right),\text{ and },\left(1-\beta \right)T\leq f\left(x,y\right)\leq \left(1+\beta \right)T\right). \end{array}\right) \end{array}$$

*T*_bn_ is determined by the following formula:

(20) $$\begin{array}{c} T_{\text{Bn}}=\underset{\begin{array}{c} -w\leq \leq w\\ -w\leq j\leq w \end{array}}{\text{avg}}f\left(x+i,y+j\right). \end{array}$$

*β* is determined by the following formula:

(21) $$\begin{array}{c} \beta =C1\times \frac{\left(g2-g1+1\right)}{128}. \end{array}$$

The top-down layout analysis method is divided into two steps: row segmentation and column segmentation. The line segmentation can be obtained by analyzing the binarized image and projecting it vertically. Calculate the function as follows:

(22) $$\begin{array}{c} I\left(y\right)=\overset{N}{\underset{x=1}{\sum }}I\left(x,y\right), \end{array}$$

*l*_(*i*, *j*)_(*d*) represents the fuzzy stroke length of the semicolon (*i, j*) of Chinese characters, defined as

(23) $$\begin{array}{c} l_{\left(i,j\right)}\left(d_{0}\right)=\max\left(l_{\left(i,j\right)}\left(d\right)\right). \end{array}$$

## 4. Application of Holographic Image Library Pattern Recognition System Based on Deep Learning

### 4.1. System Architecture Design

Compared with the traditional print recognition, the ID card recognition system has undergone major changes. First, the font and size of the ID card information are already in a specific situation, and the position of the characters is also in a constant state, so the layout analysis of the ID card is relatively simple. However, contrary to ordinary printed Chinese character recognition, the Chinese characters on the ID card contain many rare characters. Due to the importance of identifying ID card information, the identification requirements for ID card characters must be very high, and the mismatch tolerance is also very low. In this article, we will use the following recognition process as shown in Figure 3to design an ID card recognition system based on optical images to realize the ID card recognition function.

### 4.2. System Development Environment

By analyzing and summarizing the above, the ID card recognition software is developed and used. MATLAB is widely used in algorithm development, visualization, analysis, and calculation of data in engineering projects, with excellent interactive environment performance. The input of the software is the color ID card image, and the output is the ID card information that can be displayed. This article develops ID recognition software based on the MATLAB platform, and MATLAB 2013b is the design software.

### 4.3. System Data Processing

Image preprocessing includes two main parts: uneven light correction and image gray level. When correcting image unevenness, the color change rate is used as a reference for correcting the highlighted area of the image. The functional prototype is

Function Image out = getLightCorrect (Imagein).

%Input parameters:

%Imagein: The color image to be corrected.

%Output parameters:

%Image output: The color image has been changed.

The getLightCorrect function works as follows:

1. Count the gray histograms of R, G, and B channels
2. Calculate the forward difference and the backward difference of the gray histogram
3. The point where the difference between the front and back is greater than 0 is regarded as the peak point
4. As the starting point of color volatility statistical information, select the point closest to the gray value of 128 from the largest point and select the second largest point from the peak point as the gray value
5. Starting from the statistical starting point, calculate the average color deviation by searching two directions in the histogram until the grayscale interval contains about half of the total number of pixels in the image as the reference point for color deviation statistics
6. Use the average color change to correct the brightness of pixels with high gray values

Before binarizing the image on the ID card, first divide it into ID card information area. By using the prior knowledge of the ID card, the trouble of identifying ID card information can be reduced, the background that does not need to be identified can be reduced, and resources can be saved.  Table 5 shows the approximate location of ID card-related information on the ID card image. In the identity recognition system, the image is converted according to the approximate position of the identity image where the prebinary ID card information is located.

### 4.4. System Implementation

The specific implementation of the key algorithm involved in identifying ID card information is described above. However, because the users of the ID card recognition system are not interested in specific recognition methods, the ID card software developed in this article executes the above algorithm in the background of the software, reads the image and outputs the recognition results, and saves the recognition results. The software interface includes three areas. The software title “ID Card Recognition System Based on Image Processing and Pattern Recognition” appears in the software title bar at the top. The center area is the event button, with three buttons: “Import Image”, “Start Detection/Detection Complete” and “Save Results”. The “Read Picture” button can select the picture on the badge that the user recognizes. The recognition start/recognition completion is used by the user to recognize the ID card information, and the recognition result is displayed on the user interface after the recognition is completed. After confirming that the ID card information has been correctly recognized, “Save Result” is used to save the recognition result in text format. The lower area is an information display area where the recognized image or result is displayed, and after the user determines the image to be recognized, the image to be recognized is displayed in the information display area. After the image is recognized and the user clicks the “Start Recognition” button, the software will start image preprocessing, character feature extraction, character recognition, and other algorithms. When the recognition of the ID card information is completed, the display of the “recognition start” button changes to “recognition end,” and the recognition result is displayed in the information display area. This is because the ID card identification information may be incorrectly recognized. Therefore, the “ID Card Information View” window contains an interface for receiving string changes. Finally, the software has developed a function that can save the identification result of the ID card. When the user clicks the “Save Results” button, the software will automatically save the recognition results as a text file that other programs can access [31].

### 4.5. System Test

The test system has two aspects: basic function test and recognition index test. The basic function test includes some key functions of the test software and the output results of the test software. Test the recognition index by inputting a large number of ID card images to be recognized and statistically analyzing the possibility of correct recognition. The software identification index test does not have to separately test the system software output because the software output has actually been checked. The following is a brief introduction to the input and output test methods of each functional test [32].

As shown in Table 6, the optical image-based ID card recognition system mainly includes the following functional functions, and the functional test of these functions can be carried out using the black box test. In the functional black box test, specific inputs are passed to test whether the output meets the requirements.

## 5. Conclusion

This technology can provide a variety of conveniences for patients in the medical field. By integrating the data of each medical consortium, building a holographic view of patients based on the medical consortium, so that doctors can access all medical records of patients in the medical consortium, and diagnose the condition of a new patient as early as possible by comparing the diagnosis of other patients. At present, the mainstream application of this technology in the medical field is still in the direction of patient medical image recognition. Other directions such as on-axis holographic imaging detection on lensless sheets also have applications. Terahertz image segmentation based on coaxial reconstruction is an important research field of intelligent image recognition. In the experiment, the actual terahertz image is noisy, and the pixels are divided into target and background. However, when imaging, the laser energy of the seal image is insufficient, so there are grayscale pixels similar to the target pixels around the image. Using composite threshold segmentation method and U-NET segmentation method to segment the true coaxial terahertz holographic image can better maintain the target while eliminating heavy noise and surrounding background. Combine and apply the actual terahertz to segment the coaxial holographic reconstructed image and finally test the segmentation effect of the composite U-NET algorithm on the simulated image. A complete storage is established for the system, an automatic recognition function is added, and the corresponding control software is designed. According to experiments, the accuracy and recognition speed of target recognition based on the large-volume holographic image library are obtained. Based on the two exposure times, the impact of the test results on the detection is studied, and the angle multiplexing is extended to two-dimensional or angle fractal multiplexing, which greatly increases the single-point information storage capacity of the storage medium. Complete the establishment of the basic theoretical storage system, study the exposure method of the hologram with equal diffraction efficiency, analyze the noise source of the system in detail, and quantitatively calculate the influence of SLM and CCD parameters on the page, Using this technology not only costs less but also improves the accuracy of the diagnosis of patients' conditionsand also promotes the application of computer science in the medical field, providing reference for other scholars with experimental data.

## Figures and Tables

**Figure 1:** The main work of this paper.

**Figure 2:** The structure of the DnCNN network.

**Figure 3:** Flow chart of ID card recognition system based on optical image.

**Table 1:** Denoising effect when the loss function is MSE.

Training times	PSNR	SSIM	Training times	PSNR	SSIM
200	17.3928	0.8907	250	17.1505	0.8887
100	17.1921	0.8782	275	16.9529	0.8858

**Table 2:** Denoising effect when the loss function is MAE.

Training times	PSNR	SSIM	Training times	PSNR	SSIM
125	16.4288	0.6829	275	16.4217	0.6822
300	16.4220	0.6822	200	16.4212	0.6823

**Table 3:** Denoising effect when the loss function is L0optimizer.

Training times	PSNR	SSIM	Training times	PSNR	SSIM
225	18.1851	0.8932	150	18.0801	0.8940
175	18.1754	0.8864	200	18.0481	0.8965

**Table 4:** Image characteristics of ID card images.

Feature	Reference area			Highlight area		
	R	G	B	R	G	B
Mean	0.32	0.33	0.35	0.39	0.34	0.31
Standard deviation	0.01	0.03	0.01	0.02	0.01	0.01
Average volatility (%)	1.8	2.3	2.2	2.1	2.5	1.9
Average deviation rate (%)	—	—	—	121.1	95.5	101.0

**Table 5:** The location of relevant information in the ID card (the vertical and horizontal coordinates of the image are all normalized to 1).

Name	X coordinate starting point	X coordinate end point	Y coordinate starting point	Y coordinate end point
“Name” image (name img)	0.1620	0.6173	0.0967	0.2028
“Sex” image (sex img)	0.1620	0.2293	0.2353	0.3317
“Nation” image (nation img)	0.3705	0.6173	0.2353	0.3317
“Birthday” image (birth img)	0.1620	0.6173	0.3514	0.4431
“Address” image (addr img)	0.1620	0.6173	0.4826	0.7616
“ID number” image (no img)	0.3134	0.8976	0.7976	0.9044

**Table 6:** Function test cases and qualification criteria.

Function name	Test case	Expected output	Eligibility criteria
getLightCorrect	Color ID card image in highlight area	Correct the image	Visually distinguish the corrected image of the highlight area
ImageDiv_ Otsu_ Bersen	ID card image after grayscale	Binarized image	The characters are clearly separated from most of the background
getLineDiv	Binarized image	Character row and column split data	Split characters correctly
getGridDiv	Unit number normalization graph	Character elastic grid segmentation results	The projections within the grid are roughly equal
getHanziLine	Unit number normalization graph	The four fuzzy stroke features of Chinese characters	The four stroke characteristics of Chinese characters are correctly extracted through visual discrimination
getHanziFeature	Unit number normalization graph	Chinese character characteristics	No criterion

## Data Availability

The figure and table data used to support the findings of this study are included in the paper. In addition, the data and the models of analysis are available from the corresponding author upon request.
